# Efficacy of Various Types of Berries Extract for the Synthesis of ZnO Nanocomposites and Exploring Their Antimicrobial Potential for Use in Herbal Medicines

This article has been retracted.

**DOI:** 10.1155/2022/9914173

**Published:** 2022-08-16

**Authors:** Amara Dar, Rabia Rehman, Ayesha Mohyuddin, Maria Aziz, Jamil Anwar, Gashew Tadele, Noor Mohammed Kadhim, Ali H. Alamri, Rami M. Alzhrani

**Affiliations:** ^1^Centre for Analytical Chemistry, School of Chemistry, University of the Punjab, Quaid-e-Azam Campus, Lahore 54590, Pakistan; ^2^Centre for Inorganic Chemistry, School of Chemistry, University of the Punjab, Quaid-e-Azam Campus, Lahore 54590, Pakistan; ^3^Chemistry Department, University of Management & Technology, Lahore, Punjab, Pakistan; ^4^Mizan Tepi University, College of Natural and Computational Sciences, Department of Chemistry, Ethiopia; ^5^Department of Medical Instruments engineering Techniques, Al-Farahidi University, Baghdad 10021, Iraq; ^6^Department of Pharmaceutics, College of Pharmacy, King Khalid University, Abha 62529, Saudi Arabia; ^7^Department of Pharmaceutics and Industrial Pharmacy, College of Pharmacy, Taif University, P.O. Box 11099, Taif 21944, Saudi Arabia

## Abstract

Nanoscience has developed various greener approaches as an alternate method for the synthesis of nanoparticles and nanocomposites. The present study discusses the efficacy of berries extract for the synthesis of ZnO nanocomposites. Characterization of synthesized nanocomposite were done by SEM, UV/VIS spectrophotometry, Fourier transform infrared (FTIR) spectroscopy, and XRD techniques. The crystalline nature of the synthesized nanoparticles was verified by XRD pattern in the range of 10-80 nm. The UV absorption peak of *Elaeagnus umbellata* (ZnO-EU) nanocomposite at 340 nm, *Rubus idaeus* (ZnO-Ri) nanocomposite at 360 nm, and *Rubus fruticosus* (ZnO-Rf) nanocomposite at 360 nm was observed. The nanocomposites were analyzed for their antimicrobial activity and found to be effective against three phytopathogens. The antimicrobial activity of ZnO nanocomposites showed good results against *Escherichia coli* (*341*), *Staphylococcus aureus* (*345B*), and *Pseudomonas aeruginosa* (*5994 NLF*). This study presents a simple and inexpensive approach for synthesizing zinc oxide nanocomposites with effective antibacterial activity.

## 1. Introduction

Nanoscience is an advanced field of science that has brought a revolution in different areas of science like photocatalysis, medicine, chemical synthesis, and agriculture. This is mainly due to the size and morphology of synthesized materials that increase the potential applications in the said areas. Nanomaterials are called “a wonder of modern medicine” [1]. Researchers are using ecofriendly methods to synthesize different metal nanoparticles for pharmaceutical applications because of the increasing demand [2]. Nanoparticles are tiny objects which behave as a single unit in terms of properties. Nanoparticles can be classified as metal nanoparticles, nonmetal nanoparticles, semiconductor nanoparticles, nonmetal ceramic nanoparticles, and also carbon nanoparticles, based upon the type of the material used for synthesis of this single moiety [3].

Metal oxide NPs were used in different fields like soil stabilization, solar cells, biomedicine, gas sensors, wastewater treatment, and light-emitting devices [4]. Different metals have been successfully incorporated so far for the synthesis of nanoparticles and the applications of these particles has been studied in different fields. Metals like Cu, Au, Ag, Se, Ni, and Zn have been used for the synthesis of nanoparticles, and their applications in agriculture and industry have been studied. Ag has got natural tendency as an antibacterial agent, that is why it has been used in various skin ointments. Zinc oxide nanoparticles appear to be the best choice for antimicrobial activity and antibacterial activity [5]. Various plant materials are recently used for the synthesis of nanoparticles, and this approach proved an easy and low-cost method for the preparation of nanomaterials; synthesized material in turn possesses a large surface-to-volume ratio due to having small particle size, surface morphology, and size distribution [1].

Nanocomposites are composites that have at least one phase with nanometer-scale dimensions. Composite materials are synthesized to create new materials with superior qualities. In the case of metal nanocomposites, any material organic, inorganic, or polymeric can be incorporated into metals/nonmetals to synthesize the nanocomposite with tailored qualities [6]. Zinc oxide biosynthesis can be achieved with different biological materials, including fungi, plant extract, and bacteria [7].

*Elaeagnus umbellata* belongs to the family of *Elaegnaceae* and is a large shrub. It is known locally as ‘Kankoli.' It is a widespread medicinal shrub that grows wild in Azad Kashmir between 1372 and 1829 meters above sea level [8]. The purpose is to enhance the knowledge about *Elaeagnus umbellata* and to evaluate their fruits as a potential source of bioactive and antioxidant compounds [9]. *Elaeagnus umbellata* is an ornamental plant. The fruit has carotenoid lycopene, which is used against myocardial infarction and various types of cancer [10]. The fruits were included in the traditional diet because of their long-lasting application in the treatment of diarrhea, fracture, antihepatitis, and injury. The fruit is used for the preparation of foodstuffs, jams, preserves, and juices.

*Rubus idaeus* belong to the *Rosaceae* family and its common name is “Raspberry.” *Rubus idaeus* is high in vitamins, minerals, and bioactive compounds such as phenolics, anthocyanins, and organic acids. This wild fruit have a high content of vitamin C and mineral elements*. Rubus idaeus* fruit is visually appealing, delicious, juicy, and with a distinct aroma [11]. *Rubus idaeus* is well-known for its antioxidant properties. It is used to treat cardiovascular disease, diabetes, Alzheimer, cancer, and obesity [12].

*Rubus fruticosus* is a medicinal shrub that belongs to the *Rosaceae* family. *Rubus* is the largest genus in the *Rosaceae* family, with over 700 species. *Rubus fruticosus* is known by several names in different parts of the world. Its common name is “Blackberry.” *Rubus fruticosus* is a great source of phenolic compounds exhibiting antioxidant activities. *Rubus fruticosus* has a good quantity of minerals such as calcium, selenium, fluoride, iron, phosphorus, potassium, zinc, copper, and manganese. They are a good source of vitamins and minerals. These berries are consumed both fresh and processed, as they are used to make jams, syrups, and jellies [13].

In the present study, the synthesis of ZnO nanocomposites by using extracts of berries like *Elaeagnus umbellate*, *Rubus fruticosus*, and *Rubus idaeus* is a novel approach. Using plant extract in nanocomposite synthesis is a green approach that does not need sophisticated instrumentation and toxic chemicals. The use of eco-friendly harmless materials in the synthesis of ZnO nanomaterials can add many potential benefits for applications in different fields. For environmental risk management, such approach for developing material by environmentally safer route and possessing numerous benefits is highly appreciated and used in herbal and homeopathic medicines. These are usually have long-term effects and less side effects because their components are made up of natural products derived from plants. They do not have lethal effects like allopathic medicines [14–22].

## 2. Materials and Methods

Zinc acetate dihydrate (Zn(CH_3_COO)_2_·2H_2_O) was purchased from United laboratory chemicals and Sodium hydroxide from Merck.

### 2.1. Collection of Plant Material

*Elaeagnus umbellata* berries were collected in spring, and *Rubus fruticosus* and *Rubus idaeus* berries were collected in summer from Rawalakot (Azad Kashmir). The collected plant material was washed with tap water to remove dust and other impurities and finally rinsed with distilled water before the preparation of fruit extract.

### 2.2. Preparation of Fruit Extract

For the preparation of fruit extract of *Elaeagnus umbellata*, *Rubus fruticosus*, and *Rubus idaeus*, 5 g each of washed and crushed fruit was taken separately in a 250 mL borosil beaker and added 100 mL distilled water. The mixture was boiled for 10 min until the color turns reddish. The mixture was cooled at room temperature. The fruit extract was filtered by using filter paper and saved in an airtight jar for further procedure.

### 2.3. Preparation of Reagents

- Zinc acetate dihydrate solution was prepared by weighing 0.219 g of zinc acetate dihydrate and adding to it little water to dissolve, then making the volume up to mark in 50 mL measuring flask

### 2.4. Synthesis of Zinc Oxide Nanocomposites

Zinc oxide nanocomposites were synthesized by using zinc acetate dihydrate. Zinc acetate solution was added into the round bottom flask and stirred for 1 hour using a magnetic stirrer hot plate at 70°C. After this, 25 mL fruit extract was added into the solution of zinc acetate solution. The salt solution was then homogeneously combined with fruit extract of *Elaeagnus umbellata*, *Rubus fruticosus*, and *Rubus idaeus*, and gradual change in color from red to reddish-brown was observed. The mixture was covered and placed for 1 hour at room temperature. After 1 hour, the mixture was centrifuged for 12 minutes at 6000 rpm. Precipitates were dried at room temperature.  Figure 1 shows a study layout of ZnO-NCs can be obtained from fruit extracts of *Rubus fruticosus*, *Elaeagnus umbellata*, and *Rubus idaeus*.

### 2.5. Characterization of Zinc Oxide Nanocomposites

- UV/Vis analysis for synthesized nanocomposites was performed in the range of 250 to 550 nm using a double beam OPTIZEN POP UV/Vis spectrophotometer. All the three nanocomposites were analyzed in the UV/Vis region using methanol as a reference solvent, to find out the characteristic absorption value
- FTIR analysis of ZnO nanocomposites was performed in the range of 4000 to 400 cm^−1^ using Agilent Technologies Cary 630 FTIR spectrophotometer, to compare the shifts and appearance of bands in extracts and after the formation of nanocomposites
- XRD was used for the determination of the crystalline structure. Rigaku D/Max 2500 VBZ+/PC diffractometer was used for structural analysis of the nanocomposites in the range of 10° to 80°. The mean size of the crystals of zinc oxide nanocomposites synthesized from *Rubus fruticosus*, *Elaeagnus umbellata*, and *Rubus idaeus* was measured with the help of the Debye-Scherrer equation
- Surface morphology, shape, and particle size of the nanocomposites were studied by performing SEM. FEI Nova 450 Nano SEM machine was used to analyze morphology, shape, and particle size of the synthesized nanocomposites

### 2.6. Antimicrobial Activity

Clinically isolated three bacterial strains like *Escherichia coli* (*341*), *Pseudomonas aeruginosa* (*5994 NLF*), and *Staphylococcus aureus* (*345B*) were obtained from Sheikh Zayed Hospital, Lahore. These bacterial strains were selected as they are water and foodborne pathogens and degrade the quality of food and cause different diseases [23]. A small quantity of ZnO-NCs of *Elaeagnus umbellate*, *Rubus idaeus*, and *Rubus fruticosus* were dissolved in 4 mL of DMSO separately for conducting antimicrobial study. All these were then used against the bacterial strains chosen for study. Antimicrobial activity was assessed by the agar disc diffusion method. So, inoculation of testing bacterial strains was done on the agar plates with the help of swab sticks. Filter paper discs that have a diameter of about 6 mm were placed on the surface of agar with the help of sterilized tweezers. 50 *μ*L of test solutions were separately introduced on the discs and allowed to diffuse at room temperature. 50 *μ*L of DMSO was used as a negative control. Then, bacterial plates were incubated at 37°C for 24 hours. After the incubation period, inhibition zones were formed and then measured.

## 3. Results and Discussion

### 3.1. Characterization of ZnO Nanocomposites

Synthesized zinc oxide nanocomposites were characterized by Fourier transform infrared spectroscopy, X-ray powder diffraction, UV/Visible spectrophotometry, and scanning electron microscopy.

### 3.2. UV-Visible Spectroscopy

The reddish-brown precipitate obtained was dried overnight at room temperature to yield zinc oxide nanocomposites. The powder was resuspended in a 5 mL methanol solution. In Figure 2, the blue band indicates UV/VIS spectra showed an absorption maxima at 340 nm for ZnO-NCs of *Elaeagnus umbellata*, the red band indicates UV/VIS spectra showed absorption maxima at 360 nm for ZnO-NCs of *Rubus idaeus*, and the green band indicates UV/VIS spectra showed an absorption maxima at 360 nm for ZnO-NCs of *Rubus fruticosus*. Researchers have reported comparable results in previous studies [24, 25].

### 3.3. Fourier Transform Infrared (FTIR) Spectroscopy

The FTIR spectrum (Figure 3(a)) of ZnO-NCs *Elaeagnus umbellata* showed band at 3738 cm^−1^ corresponds to OH stretching vibration. The band at 2920 cm^−1^ corresponds to CH_2_ stretching vibration. The band at 2349 cm^−1^ indicates CO_2_ asymmetric stretch. The band at 1559 cm^−1^ corresponds to aromatic C=C stretching vibrations. The band appears at 1395 cm^−1^ corresponds to OH bend. The band at 840 cm^−1^ indicates C-N vibration [24].

The FTIR spectrum (Figure 3(b)) of *Elaeagnus umbellata* fruit extract shows different bands. The band at 1734 cm^−1^ corresponds to C=O stretching vibration. The band at 1317 cm^−1^ indicates C-O stretching vibration. The band at 1696 cm^−1^ corresponds to C=N vibration. The band at 1030 cm^−1^ indicates S=O vibration.

The FTIR spectrum (Figure 3(c)) of ZnO-NCs *Rubus idaeus* shows different bands. The band at 3614 cm^−1^ is attributed to OH stretching vibration. The band at 2082 cm^−1^ corresponds to the strongest C-C stretching vibration. The band at 1558 cm^−1^ corresponds to aromatic C=C stretching vibrations. The band appears at 1507 cm^−1^ corresponds to the asymmetric bending of C-H. The band at 1456 cm^−1^ indicates CH_2_ bending. The band at 1363 cm^−1^ corresponds to ZnO. The band at 959 cm^−1^ corresponds to the PO_4_ group of calcium hydroxyapatite [24].

The FTIR spectrum (Figure 3(d)) of *Rubus idaeus* fruit extract showed band at 3509 cm^−1^ indicating OH stretching vibration. The band at 1749 cm^−1^ is attributed to C=O stretching vibration. The band at 1636 cm^−1^ indicates C=C stretching vibration. The band at 1340 cm^−1^ indicates C-O vibration. The band at 653 cm^−1^ shows Cl stretching [25].

The FTIR spectrum (Figure 3(e)) of ZnO-NCs *Rubus fruticosus* shows band at 3750 cm^−1^ that corresponds to OH stretching vibration. The band at 1684 cm^−1^ corresponds to C-N stretching vibrations. The band at 1506 cm^−1^ corresponds to CO_2_ vibration. The band at 1339 cm^−1^ is attributed to aromatic C-H bend. The band at 1014 cm^−1^ corresponds to PO_4_. The band at 697 cm^−1^ confirms the formation of ZnO nanocomposites [24].

The FTIR spectrum (Figure 3(f)) of *Rubus fruticosus* fruit extract shows band at 3854 cm^−1^, which specifies OH stretching vibration. The band at 1792 cm^−1^ is attributed to C=O stretching vibration. The band at 1636 cm^−1^ indicates C=C stretching vibration. The band at 668 cm^−1^ shows Cl stretch [25].

### 3.4. Scanning Electron Microscopy

The surface morphology of ZnO-NCs of *Elaeagnus umbellata*, *Rubus idaeus*, and *Rubus fruticosus* were characterized by SEM analysis as shown in Figures 4(a)–4(c). The shape of the ZnO-NCs of *Elaeagnus umbellata* was fiber-like while for ZnO-NCs of *Rubus idaeus* was cubic-like and for ZnO-NCs of *Rubus fruticosus* was leaf-like. The particle size of the nanocomposites was calculated from ImageJ software. The average particle size of synthesized ZnO-NCs of *Elaeagnus umbellata* was 69 nm while the average particle size of synthesized ZnO-NCs of *Rubus idaeus* was 67 nm and the average particle size of synthesized ZnO-NCs of *Rubus fruticosus* was 65 nm.

### 3.5. X-Ray Diffraction (XRD)

Bragg's diffraction peaks of ZnO-NCs of *Elaeagnus umbellata*, *Rubus idaeus*, and *Rubus fruticosus*2*θ* = 31.7°, 34.3°, 36.15°, 47.25°, 56.45°, 62.75°, and 67.7° were observed by XRD spectrum. The diffraction intensities were studied from 20° to 80° at 2*θ* angles. The existence of ZnO-NCs was verified by a high-intensity broad peak at 2*θ* = 36.15° and low-intensity peak at 2*θ* = 67.7°. The mean crystallite size of obtained ZnO-NCs was verified by the Debye-Scherrer equation.  Figure 5 shows the average particle size of ZnO-NCs of *Elaeagnus umbellata* was 102.97 nm while the average particle size of ZnO-NCs of *Rubus idaeus* was 151.99 nm and the average particle size of ZnO-NCs of *Rubus fruticosus* was 102.47 nm. A similar trend is observed with ZnO/PVA nanocomposite using aqueous Moringa oleifeira leaf extract [26].

### 3.6. Antimicrobial Activity

ZnO nanocomposites synthesized by three different berries *Elaeagnus umbellata* (autumn olive), *Rubus idaeus* (raspberry), and *Rubus fruticosus* (blackberry) was assessed for their antimicrobial activity against Gram-positive *Staphylococcus aureus* (*345B*) bacteria, Gram-negative *Pseudomonas aeruginosa* (*5994 NLF*), and *Escherichia coli* (*341*) bacteria. The antimicrobial activity of ZnO nanocomposites was analyzed by the agar disc diffusion method. The presence of a zone of inhibition demonstrated the antimicrobial potential of ZnO nanocomposites.

The antimicrobial potential of ZnO-NCs of *Elaeagnus umbellata* (autumn olive), *Rubus idaeus* (raspberry), and *Rubus fruticosus* (blackberry) shows a wide spectrum of antibacterial action.  Figure 6 shows the highest zone of inhibition was identified in ZnO-NCs of *Rubus fruticosus* against *Pseudomonas aeruginosa* (*5994 NLF*) bacteria. The lowest zone of inhibition was observed in ZnO-NCs of *Elaeagnus umbellata* and *Rubus idaeus* against *Escherichia coli* (*341*) and *Staphylococcus aureus* (*345B*) bacteria, as given in Figures 7(a)–7(c). Same trend is observed with neem [27] and *Mentha longifolia* extract [28].

## 4. Conclusion

In this work, zinc oxide nanocomposites were synthesized by using the green approach. A simple method was utilized for the preparation of ZnO nanocomposite using extract of *Rubus fruticosus*, *Elaeagnus umbellata*, and *Rubus idaeus*, thereby, restricting the use of harmful chemicals for the fabrication of nanocomposites. The fruit extract was used instead of toxic reducing and stabilizing chemicals. The fabricated ZnO nanocomposites' average particle size was calculated as 102.47, 102.97, and 151.99 nm by using Debye-Scherrer's equation. Synthesized nanocomposites showed good antimicrobial potential against *Escherichia coli* (*341*), *Staphylococcus aureus* (*345B*), and *Pseudomonas aeruginosa* (*5994 NLF*) strains of bacteria.

## Figures and Tables

**Figure 1:** Synthesis of zinc oxide nanocomposites using fruit extracts.

**Figure 2:** UV/VIS spectra of *Elaeagnus umbellata* (autumn olive), *Rubus idaeus* (raspberry), and *Rubus fruticosus* (blackberry).

**Figure 3:** (a) FTIR spectrum of ZnO-NCs of *Elaeagnus umbellata* (autumn olive). (b) FTIR spectrum of *Elaeagnus umbellate* (autumn olive) fruit extract. (c) FTIR spectrum of ZnO-NCs of *Rubus idaeus* (raspberry). (d) FTIR spectrum of *Rubus idaeus* (raspberry) fruit extract. (e) FTIR spectrum of ZnO-NCs of *Rubus fruticosus* (blackberry). (f) FTIR spectrum of *Rubus fruticosus* fruit extract.

**Figure 4:** SEM image of ZnO-NCs of (a) *Elaeagnus umbellata* (autumn olive), (b) *Rubus idaeus* (raspberry), and (c) *Rubus fruticosus* (blackberry).

**Figure 5:** XRD pattern of ZnO-NCs of *Elaeagnus umbellata* (autumn olive), *Rubus idaeus* (raspberry), and *Rubus fruticosus* (blackberry).

**Figure 6:** Comparison of antimicrobial activity of zinc oxide nanocomposites of *Elaeagnus umbellata* (autumn olive), *Rubus idaeus* (raspberry), and *Rubus fruticosus* (blackberry).

**Figure 7:** Zone of inhibition of ZnO-NCs of *Elaeagnus umbellata* (autumn olive), *Rubus idaeus* (raspberry), and *Rubus fruticosus* (blackberry) against (a) *Pseudomonas aeruginosa*, (b) *Escherichia coli*, and (c) *Staphylococcus aureus.*

## Data Availability

All data related to this work are presented in Results and Discussion along with references.

## Abbreviations

SEM: Scanning electron microscopy
UV/VIS: Ultraviolet/visible spectroscopy
FTIR: Fourier transform infrared spectroscopy
XRD: X-ray diffraction
ZnO-EU: *ZnO-Elaeagnus umbellata* nanocomposite
ZnO-Ri: ZnO-*Rubus idaeus* nanocomposite
ZnO-Rf: ZnO-*Rubus fruticosus* nanocomposite
ZnO-NCs: Zinc oxide nanocomposites
EU: *Elaeagnus umbellata*
Ri: *Rubus idaeus*
Rf: *Rubus fruticosus.*
